The article "Genome Wide Linkage Study, Using a 250K SNP Map, of Plasmodium falciparum Infection and Mild Malaria Attack in a Senegalese Population" was published in 2010. Journal: PLoS One.

# Genome Wide Linkage Study, Using a 250K SNP Map, of *Plasmodium falciparum* Infection and Mild Malaria Attack in a Senegalese Population

**DOI:** 10.1371/journal.pone.0011616

**Published:** 2010-07-15

**Authors:** Jacqueline Milet, Gregory Nuel, Laurence Watier, David Courtin, Yousri Slaoui, Paul Senghor, Florence Migot-Nabias, Oumar Gaye, André Garcia

**Affiliations:** 1 UMR 216 - Mère et Enfant face aux infections tropicales, Institut de Recherche pour le Développement (IRD), Paris, France; 2 Laboratoire de parasitologie, Université Paris Descartes, Paris, France; 3 UMR CNRS 8145 - Mathématiques Appliquées Paris 5 (MAP5), Université Paris Descartes, Paris, France; 4 U 657, Institut National de la Santé et de la Recherche Médicale (INSERM), Garches, France; 5 Laboratoire de Parasitologie et de Mycologie, Département de Biologie et d'Explorations fonctionnelles, Faculté de Médecine, Université Cheikh Anta Diop, Dakar, Sénégal; Université Pierre et Marie Curie, France

## Abstract

Multiple factors are involved in the variability of host's response to *P. falciparum* infection, like the intensity and seasonality of malaria transmission, the virulence of parasite and host characteristics like age or genetic make-up. Although admitted nowadays, the involvement of host genetic factors remains unclear. Discordant results exist, even concerning the best-known malaria resistance genes that determine the structure or function of red blood cells. Here we report on a genome-wide linkage and association study for *P. falciparum* infection intensity and mild malaria attack among a Senegalese population of children and young adults from 2 to 18 years old. A high density single nucleotide polymorphisms (SNP) genome scan (Affimetrix GeneChip Human Mapping 250K-nsp) was performed for 626 individuals: i.e. 249 parents and 377 children out of the 504 ones included in the follow-up. The population belongs to a unique ethnic group and was closely followed-up during 3 years. Genome-wide linkage analyses were performed on four clinical and parasitological phenotypes and association analyses using the family based association tests (FBAT) method were carried out in regions previously linked to malaria phenotypes in literature and in the regions for which we identified a linkage peak. Analyses revealed three strongly suggestive evidences for linkage: between mild malaria attack and both the 6p25.1 and the 12q22 regions (empirical p-value = 5×10^−5^ and 9×10^−5^ respectively), and between the 20p11q11 region and the prevalence of parasite density in asymptomatic children (empirical p-value = 1.5×10^−4^). Family based association analysis pointed out one significant association between the intensity of plasmodial infection and a polymorphism located in *ARHGAP26* gene in the 5q31–q33 region (p-value = 3.7×10^−5^). This study identified three candidate regions, two of them containing genes that could point out new pathways implicated in the response to malaria infection. Furthermore, we detected one gene associated with malaria infection in the 5q31–q33 region.

## Introduction

*Plasmodium falciparum* (*P. falciparum*) malaria represents one of the most important causes of mortality and morbidity in tropical areas. Despite the strong involvement of international and national institutions to enhance the effective level of coverage of malaria interventions, the goals defined by Roll Back Malaria in 2000 seem difficult to reach [1]–[3]. However, a new general pattern is emerging, based on recent publications [4], [5], that malaria incidence is decreasing worldwide [6]. This situation stresses the necessity to pursue fundamental research activities in order to improve the understanding of malaria physiopathology, and to help to develop strategies and tools for a better control. Among the clinical presentations of malaria, asymptomatic parasitemia (i.e parasitemia without fever or any clinical sign), and mild malaria attack defined as the association of fever and parasitemia are the most frequent and have very important consequences in term of morbidity and economic effects [7], [8]. Asymptomatic parasitemia can present different aspects depending on endemicity and transmission conditions and the complexity of this phenomenon, including immune response, is not totally understood and has been recently underlined [9]. Much less frequent, severe malaria (cerebral malaria, severe anaemia and other complications) has a heavy burden in terms of mortality. Multiple factors are involved in the variability of host's response to infection, like the intensity and seasonality of malaria transmission, the virulence of parasite, which could depend on its genetic polymorphism, and host characteristics like age or genetic make-up. Although admitted nowadays, the involvement of host genetic factors remains unclear [10]. Discordant results exist, even concerning the best-known malaria resistance genes that determine the structure or function of red blood cells [11], [12].

The great majority of genetic epidemiology studies used candidate genes approach which is restricted to the examination of specific genes, based on their presumed functional relevance to malaria (e.g. genes involved in the control of immunity). These studies led to numerous but frequently discordant results. For example association between polymorphisms within the Major Histocompatibility Complex (MHC) region on chromosome 6p21–p23, that contains the Tumor Necrosis Factor alpha (TNF-α) gene, and severe [13]–[17] but also mild malaria [18], [19] has been demonstrated in several population in particular in Gambian children. However, discordant results exist concerning the involvement of TNF-α promoter polymorphisms that has been confirmed neither in Kenya [17], [20] nor in Mali [21]. The same pattern of discrepancy was observed for a polymorphism of the gene encoding IL-10 that has been shown associated with severe malaria in a population based study but not confirmed in family data [22]. Concerning asymptomatic mean parasite density Garcia et al. [23] showed the involvement of the 5q31–q33 chromosomal region in a Cameroonian population and this result was rapidly confirmed in another area by Rihet et al. [24]. Many reasons can explain these discrepancies, such as the diversity of phenotypes definition, the level of malaria transmission and the way by which they are taken into account. Furthermore, genetic heterogeneity between populations, gene-environment interactions or epistasis can play an important role. Previous studies focused also essentially on genes involved in the control of immunity although a lot of unknown factors could contribute to the physiopathology. Indeed current estimate shows that genetic host factors account for approximately 25% of the total variability in malaria incidence when the strongest genetic effect known until now (hemoglobin S) explains only 2% [10]. The complexity of this genetic control, and the role of malaria as one of the major driving forces for genetic selection have been underlined in recent reviews [25], [26]. In this sense approaches such as genome-wide studies that allow studying the role of hundreds of thousands single nucleotide polymorphisms (SNPs) as genetic markers without specific functional hypotheses [27] could help understanding the complexity of the disease by identifying new genes.

To our knowledge three genome wide studies have been performed in malaria area [11], [28], [29], one of them concerning severe malaria [11]. They showed discordant results too. The first one, performed in a rural population from Ghana, was based on 10,000 single-nucleotide polymorphisms. This study showed a prominent signal on chromosome 10p15 obtained with malaria fever episodes and a borderline non significant trend on chromosomes 13q and 1p36 with parasite density and anaemia respectively [29]. In opposite no signal of linkage were obtained in 5q31q33 or 6p (MHC) region. The second genome wide linkage study was performed in a Senegalese population and used 400 microsatellites as markers. This last study confirmed the linkage between 5q31 region and asymptomatic parasite density, whereas suggestive linkages were identified between three additional regions: 5p15, 13q13 for malaria attack and 12q21 for the maximum parasite density during asymptomatic infection [28]. The third genome wide study, concerning severe malaria, pointed out above all the considerable genetic diversity between populations in Africa and the weak level of linkage disequilibrium existing between SNPs markers compare to European populations [11].

Here we report on a genome-wide linkage study for *P. falciparum* infection intensity and mild malaria attack among a Senegalese population of children. The population belongs to a unique ethnic group and was closely followed up during 3 years. Genotyping of SNPs was performed using the high density Affimetrix GeneChip Human Mapping 250K-nsp (262,264 SNPs).

## Results

### Phenotypes

Individuals included in the follow-up were aged from 2 to 18 years at the beginning of the study (mean age (SD) = 8.97 years (3.57)). Four children with less than 8 thick blood smears (TBS) during the follow-up were excluded from analyses. Other children had on average 14 TBS. Distribution of raw data and final phenotypes are presented on Figure 1. The mean rate of positive blood smears (SD) per child was 0.42 (0.18) during the follow-up. The number of mild malaria attacks ranged from zero to six and 52% of children experienced at least one malaria attack.

**Figure 1:** Distribution of raw data and phenotypes of analysis sample (372 children). (Ai to Di) Raw data. (Ai) Mean of the whole parasite density values per children. (Bi) Mean of parasite density values per children considering only positive thick blood smears. (Ci) Rate of positive thick blood smears per child during the follow-up. (Di) Total number of mild clinical malaria attacks experienced per children during the active clinical survey. (Aii to Dii) Phenotypes. (Aii) Mean level of *P.falciparum* density. (Bii) Intensity of *P.falciparum* infection. (Cii) Prevalence of *P.falciparum* infection. (Dii) Mild Malaria Attack.

Statistical approaches used to define phenotypes and the correlations between phenotypes are summarized in Table 1. All phenotypes were adjusted on age except PrevPI (p-value = 0.74). We didn't observe any decrease of positives blood smears rate with age. The only other covariates included in final models for asymptomatic infection were the follow-up year (1^st^, 2^nd^ or 3^rd^ year), consistent with a different transmission level between the 3 years, and the transmission season. HbS and G6PD polymorphisms had no effect on MLPD, IntPI and PrevPI phenotypes but we observed a strong effect of HbS polymorphism (p = 3.56×10^−6^) on MMA phenotype. Note that no effect of sex or village was detected on any of the phenotypes. From 364 to 370 children were genotyped, depending on phenotype, and included in linkage analyses. The estimations of heritability were 0.08, 0.26, 0.26 and 0.40 respectively for MLPD, IntPI, PrevPI and MMA.

**Table 1:** Definition of phenotypes related to *P. falciparum* infection or morbidity.

Phenotype$	Selection criteria	Statistical Method	Significant covariates	Correlations		
				MMA	MLPD	IntPI
**MLPD**	≥8 blood smears	Mean of LPD adjusted for covariates using a linear regression model	Age (p = 0.0014); Visit (p<10^−4^)	r = −0.001 (p = 0.98)		
**IntPI**	≥8 blood smears; at least one positive blood smear	Linear model with mixed effect	Age (p<10^−4^); Follow-up year (p = 0.0003); Season (dry/rainy, p<10^−4^)	r = 0.20 (p<10^−4^)	r = 0.59 (p<10^−4^)	
**PrevPI**	≥8 blood smears	Logistic regression model with mixed effect	Follow-up year (p<10^−4^); Season (dry/rainy, p<10^−4^)	r = −0.19 (p<10^−4^)	r = 0.78 (p<10^−4^)	r = 0.02 (p = 0.97)
**MMA**	HbS polymorphism genotyped	Poisson regression model	Age (p<10^−6^); HbS (p<10^−5^)			

$ MMA, Mild Malaria Attack; MLDP, Mean Level of *P. falciparum* Density; PrevPI, Prevalence of asymptomatic *P. falciparum* Infection; IntPI, Intensity of *P. falciparum* Infection.

Abbrevation: LPD, log transformed values of parasite density.

### Linkage analysis

The variance component (VC) and regression-based (RB) linkage analysis were applied to the data. Results for RB analysis are shown in Figure 2 and 3 and main linkage results are summarized in Table 2.

**Figure 2:** Results of quantitative multipoint linkage analysis obtained from the regress-based method implemented in MERLIN program for chromosomes 1–12. Genetic position (cM) is plotted along the x axis. The dotted line indicates the LOD score associated with the threshold p-value of 10^−3^ and the dashed-dotted line the LOD score associated the threshold p-value of 10^−4^.

**Figure 3:** Results of quantitative multipoint linkage analysis obtained from the regress-based method implemented in MERLIN program for chromosomes 13–22 and pseudo-autosomal region of chromosome X. Genetic position (cM) is plotted along the x axis. The dotted line indicates the LOD score associated with the threshold p-value of 10^−3^ and the dashed-dotted line the LOD score associated the threshold p-value of 10^−4^.

**Table 2:** Chromosome regions with a genome-wide suggestive LOD score.

Phenotype$	Region	SNP/cluster	Physical position	RB method LOD score	RB method 1-LOD support interval	No. of GW peaks*	Functional candidate genes£
**MMA**	6p25.1	rs4959312	4,646,134	3.50	4,504 Kb–5,864 Kb	0.08	*LYRM4*
**MMA**	12q22	rs4275668 to rs10777556	92,809,721	3.49	91,951 Kb–93,132 Kb	0.08	*PLXNC1*, *UBE2N*, *SOCS2*
**PrevPI**	20p11q11	rs6138473 to rs2073077	24,959,423	3.58	23,839 Kb–33,378 Kb	0.09	*PROCR*, *RIN2*, *RBBP9*, *HCK*, *BCL2L1*, *CST7*
**MLPD**	20p11q11	rs6138473 to rs2073077	24,959,423	3.63	17,285 Kb–30,788 Kb	0.15	*PROCR*, *RIN2*, *RBBP9*, *HCK*, *BCL2L1*, *CST7*
**IntPI**	9q34	rs10819510	131,195,485	3.08	131,076 Kb–132,010 Kb	0.14	*ASB6*

$ MMA, Mild Malaria Attack; MLDP, Mean Level of *P. falciparum* Density; PrevPI, Prevalence of asymptomatic *P. falciparum* Infection; IntPI, Intensity of *P. falciparum* Infection.

* Number of peak expected by chance per genome scan.

£ LYRM4, LYR motif containing 4; PLXNC1, plexin C1; UBE2N, ubiquitin-conjugating enzyme E2N; SOCS2, suppressor of cytokine signaling 2; PROCR, protein C receptor, endothelial; RIN2, Ras and Rab interactor 2; RBBP9, retinoblastoma binding protein 9; HCK, hemopoietic cell kinase; BCL2L1, BCL2-like 1; CST7, cystatin F (leukocystatin); ASB6, ankyrin repeat and SOCS box-containing 6.

Abreviation: LOD, logarithm of odds; GW, genome-wide.

Two evidence of linkage signals were obtained for MMA. The first one on chromosome 6p25.1 showed a logarithm of odds (LOD) score of 3.50 (empirical p-value = 5.0×10^−5^) and 3.96 (empirical p-value = 1.1×10^−4^) for RB and VC respectively. According to Lander and Kruglyak [30] this linkage signal can be considered as strongly suggestive since simulations showed this peak to be nearly genome-wide significant (average number of peak per replicate = 0.08 for RB analysis). The maximum asymptotic LOD score with RB was located at marker rs4959312 corresponding to 12.13cM (4.6Mb). The 1-LOD support interval defined a 3.14cM/1.3Mb chromosomal distance (from SNP rs84996 to cluster rs9504552/rs9378995) containing 12 genes. Among them *LYRM4* (LYR motif containing 4) interacts as an adaptor between frataxin and NFS1/ISCU, an essential component of iron-sulfur cluster biogenesis that could connect with immune response.

The second region with evidence of linkage for MMA phenotype was obtained on chromosome 12q22 with a LOD score of 3.49 (empirical p-value = 9.0×10^−5^) and 3.40 (empirical p-value = 3.0×10^−4^) for RB and VC respectively. In this case too, the linkage signal can be considered as strongly suggestive (average number of peak per replicate = 0.08 for both RB and VC analyses). The maximum asymptotic LOD score with RB was located at a cluster of markers from rs4275668 to rs10777556 corresponding to 104.11cM (92.8Mb). The 1-LOD support interval defined a 1.34cM/1.18Mb chromosomal distance (from rs4590917/rs10859418 to rs11107437/rs7316309) containing 12 genes as well. Several ones can be considered as functional candidates: *PLXNC1* (Plexin C1) involved in the up regulation of ICAM1 (intercellular adhesion molecule 1); *UBE2N* (Ubiquitin-Conjugating Enzyme E2N) involved in cytokine signalling pathways (MAPK and IKK) directly implicated in the modulation of immune response [31]–[33]; *SOCS2* (Suppressor of Cytokine Signaling 2) involved in the control of the proinflammatory cytokines production [34].

For asymptomatic infection, evidence of linkage was obtained for the phenotype prevalence of infection (PrevPI) on chromosome 20p11q11 with a LOD score of 3.58 (empirical p-value = 1.5×10^−4^) and 2.78 (empirical p-value = 1.6×10^−4^) for RB and VC respectively. This linkage signal is highly suggestive as well since average number of peak per replicate was 0.09 for RB analysis. Interestingly the same chromosomal region showed a suggestive linkage signal with the phenotype MLPD with a LOD score of 3.63 (empirical p-value = 1.2×10^−4^) and 2.20 (nominal p-value = 0.0011) for RB and VC analyses respectively (average number of peak per replicate = 0.15 for RB analysis). For both phenotypes, the maximum asymptotic LOD with RB was located at a cluster of markers from rs6138473 to rs2073077 corresponding to 54.76cM (24.96Mb). The 1-LOD support interval encompassed an 11.44cM/13.5Mb, and a 3.33cM/9.5Mb chromosomal distance for respectively the PrevPI and MLPD phenotypes. The first region contains 149 genes and the second one 129. Possible functional candidates include the following genes: *PROCR* that could interact in an immunomodulatory process; *RIN2* encoding a small GTPase involved in membrane trafficking in the early endocytic pathway that can reduce the endothelial integrity; *HCK* encoding a tyrosine kinase that could play a role in nitric oxide and TNF alpha secretion in macrophages [35]; *DEFB123*, belonging to a beta-defensin gene family that play a role in innate immunity [36].

Finally, a suggestive linkage signal was obtained with the 9q34 chromosomal region for IntPI phenotype, showing a LOD score of 3.08 (empirical p-value = 1.4×10^−4^) and 1.63 (empirical p-value = 0.0011) for RB and VC respectively (average number of peak per replicate = 0.14 for RB analysis). The maximum LOD score was achieved for rs10819510, corresponding to 137.7cM/131.19Mb. The 1-LOD support interval encompassed a 2.55cM/933Kb chromosomal distance, containing 18 genes. Among them, *ASB6* (for ankyrin repeat and SOCS box-containing 6) could constitute a candidate gene. The other genes in this region seem not to be involved either in immune response or in red blood cell physiology.

Analyses within these four regions using a subset of SNPs in linkage equilibrium identified by MASEL algorithm, gave very similar results indicating that the linkage disequilibrium (LD) between SNPs is taken into proper account by the method implemented in MERLIN.

### Family based association analysis

Finally, to explore the chromosomal regions we identified during linkage analysis (6p25.1, 12q22, 9q34 and 20p11q11) but also the 5q31q33 and 10p15 regions, which have been described as involved in the control of parasitemia and malaria fever episodes respectively [23], [29], we performed a linkage and association study using family based association tests (FBAT) software. For MMA, association was tested within 6p25.1, 12q22 and 10p15 regions. For each phenotype of *P. falciparum* density (PD), association was tested with the 5q31q33 region and respectively, with the 9q34 region for IntPI, and the 20p11q11 for both PrevPI and MLPD. From 1339 to 2062 SNPs were tested per phenotype. Following Li and Ji procedure [37] these subsets of SNPs were equivalent to 833, 1209, 1344, and 1626 independent tests for respectively MMA, IntPI, PrevPI and MLDP.

Taking into account multiple testing, no linkage/association was found within the regions we identified in this study neither within 10p15 region. In contrast a significant association and linkage was found in 5q31.3 region between the phenotype IntPI and SNP rs830532 located in *ARHGAP26* gene (uncorrected p-value = 3.7×10^−5^ and corrected p-value = 0.045). *ARHGAP26* (Rho GTPase activating protein 26) codes for a protein acting in particular as a negative regulator of Rho A. It is interesting to note that even non significant, a borderline association and linkage evidence to MLPD (uncorrected p-value = 8.5×10^−4^) was observed for a SNP (rs1056189) located in 5q31.1 region within a gene which has also been proposed to participate in the regulation of Rho proteins (*FLJ41603*).

Haplotypes analyses (results not shown) did not improve the results obtained with single SNP association.

## Discussion

To our knowledge, this is the first genome-wide study applied to non severe malaria that used a high density GeneChip array. We identified three strongly suggestive evidences for linkage: between mild malaria attack and both the 6p25.1 and the 12q22 regions, and between the 20p11q11 region and the prevalence of parasite density in asymptomatic children (PrevPI). Although not strictly significant, our linkage peaks are located in chromosomal regions containing relevant candidate genes involved in the control of immunity. The more relevant ones will be presented latter in the discussion. Suggestive linkages were also shown between the mean level of non zero PD measurements (IntPI) and the 9q34, and between the Mean Level of P. falciparum Density (MLDP) and the 20p11q11, regions respectively. The family based association analysis pointed out one significant association between the intensity of plasmodial infection (IntPI) and a polymorphism located in *ARHGAP26* gene in the 5q31–q33 region.

Our study was originally designed for a genome-wide linkage analysis. The high density SNPs map used here allows to provide higher information content compared to microsatellite maps and to define smaller intervals around linkage peaks. Furthermore our family sample allows us to perform an association analysis as well, which provides non-redundant and complementary information. In linkage analysis with dense SNP maps particular attention must be paid to the LD between SNPs, because it can be responsible for a bias. To deal with this point, we used the method implemented in Merlin which performs well in our particular case: relatively few parents missing and a low LD between markers. However this low LD characteristic of African populations constitutes in counterpart a handicap for association analysis. As LD between SNPs and causal variants are lower in African than in European populations, it is more difficult to achieve significant threshold for association analysis [11]. A 250K map is surely not dense enough to screen accurately candidate regions however it enabled us to detect one significant associated SNP in 5q31q33 region.

Several environmental and behavioural factors, that can be shared by groups of individuals within (or not) families, can influence both the risk of disease and the response to infection [38]. These factors have to be taken into account during the survey in order to stratify or to adjust for during analyses.

Among these factors, a very particular attention must be paid for transmission intensity and anti-malaria medicine intake. Data on transmission level in Niakhar area are consistent with a strong homogeneity of transmission rates [39] and we performed mosquitoes catching during the follow-up that confirmed this homogeneity. Furthermore, during the first year of this follow-up, we compared the mean parasite densities in 999 children living in 17 hamlets of the same villages. We found no geographical differences between the mean levels of infection within the area, consistent with the hypothesis of homogeneity [38]. Lastly, the very low utilisation of bed net (e.g. 5.7% of children) is also a statement for a weak variability of the probability to be infected during the three years follow-up.

Medicine intake was taken into account because the children received their treatment within our research program framework. Nevertheless, it is well known that despite the intensive presence of health workers in area (see www.ird.sn/activites/niakhar/), uncontrolled circulation of drugs existed and, at this time, concerned essentially chloroquine [40]. However, we performed repeated controls for the presence of chloroquine and its metabolites in urine. At each control, the presence of chloroquine metabolites in urine had no significant effect on the parasite density determined at the same moment, consistent with the high level of resistance to chloroquine in the area.

Malnutrition, co-infection and general health status of the population under study are additional limitations to accurately determine phenotypes. Indeed although discordances exist concerning the risk to develop malaria in the presence of helminth coinfection [41], [42], [43], a recent study showed that the presence of helminth infection modulates the immune response to malaria parasites, and could interfere with gene expression [44]. Obviously, nutritional status could also be responsible for the variability of malaria related morbidity and specific immune response [45], [46]. These aspects are probably a weakness of our study design and of the other genetic analysis studies of malaria. However, inclusion of all these potential confounding factors would represent a very complex study design, all the more that the duration of the survey is long and all these characteristics probably change with age.

In our study children harbouring G6PD and HbS polymorphisms were included in analyses and the potential effects of these polymorphisms were accounted for. Concerning this particular point in Ghana [29] any individuals with any of the major haemoglobinopathies were excluded from analyses whereas Sakunthabai et al. [28], in Senegal, like in our study realised the analysis on the whole population. Although this difference of sampling can contribute to the discrepancy between results, the intrinsic complexity of the red blood cells polymorphisms must clearly be considered as the principal reason. As an example, it has been highlighted that epistatic interaction between these polymorphisms can influence the protective effects of each of them [47]. Interactions of this sort are unpredictable and, if common, could make the hunt for both protective alleles and their mechanisms even more difficult.

Our study shows very little overlap with the preceding genome-wide linkage studies. However for all the regions identified by genome scan except one (10p15), linkage did not reach statistical significance. The discrepancy between results could be also explained by parasite genetic variability and/or by the genetic heterogeneity in the susceptibility/resistance mechanisms to malaria in host. About this last hypothesis it is interesting to note that the only result in common with other studies is the evidence of linkage in 12q22 region. This region is located close (1.5 Mb) to the linkage peak obtained by Sakuntabhai *et al* at marker D12S351 (12q21). This linkage is detected for two different phenotypes, malaria attacks in our study, the maximum of PD in Skuntabhai *et al.*, but in two neighbouring Senegalese populations.

Among the regions identified in this linkage analysis, two of them can be considered particularly interesting because they contain genes involved in pathways related to immunity, the 12q22 and the 6p25.1 ones.

In 12q22 region we noticed three candidate genes. *PLXNC1* encodes plexin C1 (VESPR/CD232), one of the receptors of semaphorins which are a large family of secreted and transmembrane signalling proteins (review in Mizui et al. [48]). It is now becoming clear that several semaphorins, in particular the transmembrane ones, are involved in immune response [49] and Plexin C1 was found to interact with several semaphorins on monocytes [50], [51]. It has been demonstrated that exposure of monocytes or immature dendritic cells to soluble SEMA4D/CD100, the first semaphorin characterized within the immune system, resulted in a significant down-modulation of proinflammatory cytokine production [52]. Interestingly, another class of semaphorin binds to plexinC1 and induces aggregation, cytokine production, but also surface expression of ICAM-1 [51] an immunoglobulin-like cell adhesion molecule that plays an important role in the binding of *P. falciparum* infected erythrocytes to the vascular endothelium. A second candidate gene *UBE2N* is also strongly implicated in the regulation of immunity. In mice with B cell-specific deletion of *UBE2N*, Yamamoto et al [53] demonstrated an impairment of humoral immunity. In human, the product of this gene, together with other molecules, interacts with CD40 resulting in a broad variety of immune and inflammatory responses including T cell-dependent immunoglobulin class switching and memory B cell development. These complex cellular processes involve MAPK and IKK signalling pathways that can lead to enhance natural killer cells activity and induce the differentiation and maturation of CD3, CD4, CD8 and dendritic cells, and interact with Toll-like Receptors [54], [55]. The third candidate gene from this region *SOCS2* (or *STAT2* for signal transducer and activator of transcription 2) is also strongly related to the control of immunity. Indeed, SOCS proteins negatively regulate receptor signalling via the Janus kinase/signal transducer and activation of transcription pathway (JAK/STAT pathway) [56]. In mouse model, Machado et al. [34] demonstrated that *SOCS2* deficient mice had, during intracellular infection, uncontrolled production of proinflammatory cytokines, aberrant leukocyte infiltration and elevated mortality. Very recently, the differential roles of some SOCS proteins during coinfection with *P. falciparum* and helminth in children have been shown [44]. Kim et al., [57] showed that genes encoding STAT1 and STAT2, which transmit signals from interferon receptors and are upregulated by interferon and increased in relative mRNA abundance in response to *P. chabaudi* infection. Consistent with *STAT1* and *STAT2* activation, they also observed an increased abundance of genes encoding downstream targets of interferon signalling in response to infection, including the interferon regulatory factor 1 gene, located in the 5q31q33 chromosomal region. It is also interesting to note that another member of STAT family (i.e. STAT6) could be involved in mediating erythropoietic suppression during acute blood-stage malaria and that interleukin-4 (in 5q31–q33 region) and possibly interferon-γ could also play a role in this mechanism [58].

6p25.1 chromosomal region contains a gene involved in iron-sulfur (Fe-S) cluster biogenesis (i.e. *LYRM4*). The product of this gene interacts with the cystein desulfurase (Nfs1) and its scaffold protein (IscU), and is required for the initial step of Fe-S cluster assembly. Fe-S clusters are involved in multiple cellular processes, including macrophages activity. It has been demonstrated that Nfs1 and IscU were strongly down-regulated at both mRNA and protein levels in IFN-γ stimulated macrophages. As immune response against *P. falciparum* infection is initiated by early interferon response, these data suggest a connection between the immune responses and the biogenesis of Fe-S clusters [59].

In the present study, no evidence of linkage was obtained for parasite density to the 5q31–q33 chromosomal region but we demonstrated a significant association between the intensity of plasmodial infection (IntPI) and a polymorphism located in *ARHGAP26* gene in 5q33.1 region. These results are not inconsistent since information used by both analyses (i.e. linkage and family-based association tests) are different [60].

We were the first group to underline the potential interest of this chromosomal region in a small sample of 9 Cameroonian nuclear families by detecting a borderline significant linkage between the mean level of *P. falciparum* density and the D5S636 marker [23]. This linkage was rapidly replicated by Rihet et al. [24] in Burkina Faso (marker D5S658) while Flori et al. [18] identified a linkage at the same marker D5S636 in a second population in Burkina Faso and an association with one marker (D5S487) within the 5q33.3 region. Sakuntabhai et al. [28] observed a linkage near marker D5S436 with the mean parasite density in the population of Dielmo in Senegal. All these studies concluded to the importance of this chromosomal region for two main reasons. Firstly, this region contains a cluster of genes encoding for Interleukins (*IL3*, *IL4*, *IL5*, *IL9* and *IL12B*) and for other genes involved in immunity: *IRF1* for immune regulatory factor 1; *CSF2* for colony stimulating factor 2; *c-fms*, the gene encoding the receptor of the colony-stimulating factor 1 (CSF1R). Secondly, linkage between the 5q31 locus and other parasitic diseases, such as schistosomiasis [61] and leishmaniasis [62] has been identified, as well as other immune related disorders including asthma [63].

Nevertheless, previous studies did not allow identifying the causative gene(s) and variant(s) possibly involved in this complex control. The SNP identified here (i.e. rs830532) is located in the 5q33.1 region, where are located the three markers for which the linkage with the intensity of infection was demonstrated (D5S636, D5S658, D5436). We did not regenotype this SNP to discard possible genotyping errors and confirm our result. Anyway it seems unlikely that genotyping errors occurred systematically according to the phenotype IntPI and then bias our result in favour of association [64]. Furthermore we compared the LD around the SNP rs830532 in the Hapmap Yoruba sample and in our population (data not shown) and found a very similar pattern of LD, in particular a block of high LD of 3 SNPs containing rs830532. This SNP is located in a gene, *ARHGAP26*, which is involved in the integrin signalling transduction pathway. Although the role of cytoadherence in malaria is clearly admitted, little is known of signalling triggered by this cytoadherence. The protein encoded by *ARHGAP26* acts as a negative regulator of RhoA, a member of Rho family, which cooperates in Rho kinase pathways that reduce the endothelial integrity, and is activated by the adhesion of *P. falciparum* to endothelial cells *in vitro*. Members of the Rho family are known to play an important role in the signal transmission of various receptors, including ICAM-1, one of the endothelial receptors of *P. falciparum* infected erythrocytes. The importance of the integrity of endothelial cells [65] and of the Rho kinase pathway [66] underlies the potential interest of *ARHGAP26* as a functional candidate gene.

All together, this work underlines several chromosomal regions which could play a role in resistance mechanism to malaria infection: 12q22 which have already been pointed out by a previous linkage analysis and three new regions (6p25.1, 20p11q11 and 9q34). Two of them contain very few candidate genes and, if confirmed in association analysis, could point out new pathways implicated in the response to malaria infection.

## Materials and Methods

### Study population and area

The study took place in the Niakhar area located 150 km south-east from Dakar, the capital city. Niakhar area is composed of 30 villages, regrouping 30,000 persons, the great majority of them belonging to the Sereer ethnic group. Malaria is endemic in the area and its transmission is seasonal and estimated between 9 and 12 infective bites per person per year, occurring almost exclusively between September and December, following the rainy season from July to September. Transmission is due exclusively to the complex *An. gambiae s.l.* of which 97% were represented by *An. Arabiensis* [39]. Mosquito catches performed during the follow-up (i.e. in 2002 and 2003) confirmed a homogeneous distribution of malaria vectors in the study villages (unpublished data).

Two villages of the area (Diohine and Toucar) were included in the study because of the existence of a dispensary with which we collaborated for several years. In January 2001, 1,202 children and young adults from 2 to 18 years old lived in these villages. A cohort of 504 individuals living with their two parents, and who agreed to take part in our study (informed consent signed by parents) was constituted. Neither age nor sex differed significantly between children included and not included in the cohort (p-value >0.18 and p-value >0.08 respectively).

### Clinical and parasitological survey

A TBS was collected to measure the PD in June, September, November and December 2001, in January, June, September, October and November 2002 and in January, April, June, September, October and December 2003. TBS were stained with Giemsa and asexual parasites (*P. falciparum*; *P. malariae* and *P. ovale*) and leucocytes were counted. The PD was defined as the number of parasites per 100 leucocytes. This mode of calculation allowed avoiding misestimations of the parasitemia resulting from its determination on the basis of an assumed count of white blood cells per microliter of blood [67]. A TBS was declared negative when no parasite was detected in 200 fields.

Additionally, an active clinical survey aimed at detecting any malaria attack was performed during 2002 and 2003. The children were visited twice a week by trained primary health agents to check temperature and to ask for any clinical health problem that may occur. The parents were invited to bring the child with fever or history of fever to the dispensary. In case of presumptive malaria, a TBS was performed and a questionnaire concerning clinical signs and previous treatment was filled out. Children were treated according to the recommendations of the Senegalese National Control Program for malaria. Children were considered as suffering from a mild clinical malaria attack when axillary temperature was greater or equal to 37.5°C (or reported history of fever between two systematic surveys) with a PD above 2500 trophozoites/µL. We only considered malaria attacks due to *P. falciparum*. Children had a free access to health services, whatever the reason, and the research program took care of all the treatments.

All participants were recruited, and human experimentations were conducted, in Senegal. This protocol was previously submitted and accepted by the ethic committee of the Health Minister of Senegal (N° 000526/MS/DERF/DER). At the time the study took place, all the programmes managed by the Unite de Recherche 010 from the Institut de Recherche pour le Développement in Senegal followed this procedure. We obtained informed consent from all participants involved in our study. This consent was written, translated in Serer, and obtained from all the families included in the study.

### Individual, behavioural and environmental risk factors

For each child the following information was collected: (1) age (in years); (2) sex; (3) ethnic group (all children were from the Sereer group); (4) village of residence. We also noticed the presence of co-infection with *P. malariae* since co-infections could influence the level of PDs [68].

Malaria infection can be influenced by variation in exposition to mosquito's bites as well as by prophylaxis intake. In the cohort 29 children (5.7%) declared the use of a bed net during the preceding night (validated only if the mosquito net was seen by the investigator). Neither the measurements of *P. falciparum* asymptomatic infection nor MMA (*cf. infra* in the phenotype definition section) differed significantly (p>0.10) between children declaring to use a bed net and other children. Two ways were used to take into account medicine intake. Firstly, if a child was treated, by our team, for malaria attack during the follow-up, his PD measurement was not included in the mean level of *P. falciparum* infection during the following three weeks. Secondly, although most of the time children received their treatment within our research program framework, the uncontrolled circulation of drugs in Niakhar remains an important problem (essentially chloroquine in this area [40]). To deal with this uncontrolled medicine intake, urine samples were collected 12 times during the follow-up to control for the presence of chloroquine and its metabolites in urine [69]. At each control, the presence of chloroquine metabolites in urine had no significant effect on the PD determined at the same moment. Both medicine intake and use of bed net were not included in further analyses.

### Phenotypes definitions

We were interested by asymptomatic *P. falciparum* infection and mild malaria disease. Concerning asymptomatic infection we defined three phenotypes of interest: (1) the mean level of *P. falciparum* density (MLPD) taking into account all the measurements performed during the follow-up, including negative TBS. This mean parasite density correspond to the phenotype for which the 5q31q33 chromosomal region were initially described [23], [24]; (2) the intensity of asymptomatic *P. falciparum* infection (IntPI) that took into account only the positive TBS during the follow-up. This phenotype emphasizes the ability of an individual to tolerate parasite density without clinical disease; (3) the prevalence of asymptomatic *P. falciparum* infection (PrevPI). This prevalence reflects the acquisition of a non-sterilising immunity, occurring after repeated infections, but also dependent on human genetic factors involved in immune control, and acting independently of exposure. Analyses were realised on log transformed PD values (LDP) using log (PD+1) transformation to allow for 0 count. As some children may have not been present at each visit, we considered only the children with at least height measurements out of the fifteen performed during the follow-up.

#### Mean level of *P. falciparum* density (MLPD)

We used the same statistical method as in Garcia et al. [23] to compute this phenotype in order to compare the results of the present study with our previous ones that allowed identifying the 5q31–q33 chromosomal region as involved in the control of the level of *P. falciparum* infection. To deal with a unique variable accounting for the intensity of malaria infection, a mean log parasite density was computed for each subject, based on all their TBS, positive or negative. During the follow-up, the LPD varied significantly with time (p-value <10^−4^) consistent with the variation of malaria transmission. Then, before computing the mean level of infection, individual LPD were adjusted for this variability, by subtracting the mean LPD of the corresponding visit. Once computed, the mean level of infection was adjusted for the other risk factors (age, co-infection by *P. malariae…*) using a multiple linear regression. MLPD corresponds to the residual of the multiple linear regression, and was referred as the mean level of *P. falciparum* density during the follow-up.

#### Intensity of *P. falciparum* infection (IntPI)

The intensity of parasite infection was obtained through a linear model with mixed effect. We only considered here positive measurements (thus we excluded a total of 7 individuals with no positive thick blood smear). A stepwise model selection leaded to adjust for fixed effects (age, season, co-infection with *P. malariae*, year, sex and village) as well as one random intercept per individual in order to take into account the repeated measurements. We associated a residual density to each individual by considering the normalized sum of the model residuals (each measurement residual being the difference between the response variable and the fixed effects prediction of the model) for each individual.

#### Prevalence of *P. falciparum* infection (PrevPI)

For the prevalence, the residual risk of having a positive blood smear was estimated through a logistic regression model with mixed effect, to take into account repeated measurements. A classical stepwise model selection leaded to adjust for several fixed effect (age, season, co-infection with *P. malariae*, year, sex and village) as well as one random intercept per individual in order to take into account the repeated measurements. A Pearson residual was then derived for each individual by considering the normalized difference between the observed and expected number of positive blood smear for each individuals (each measurement contribution being the inverse logit of the fixed effects part of the model).

#### Mild Malaria Attack (MMA)

The total number of mild clinical malaria attacks experienced per children during the active clinical survey was adjusted for predefined covariates using a Poisson regression model. The effects of covariates in the model were assessed using a sandwich estimator. Finally, the phenotype was obtained by calculating residuals from the Poisson regression model.

### Genotyping

Venous blood samples of 5 ml were obtained at the end of the follow-up from children and parents.

The genetic variants of Hemoglobin HbS and glucose-6-phosphate-dehydrogenase (G6PD) deficiency A- were determined on children. Frequencies of these variants in this Sereer ethnic group are 0.13 for HbS and 0.16 for G6PD A- [70]. Effect of these genetic factors on phenotypes was taken into account by including them as covariates in the models defined above. For G6PD, girls heterozygous and homozygous for the variant A- were pooled together.

Overall, a high density SNP genome scan was performed for 626 individuals: i.e. 249 parents and 377 children out of the 504 ones included in the follow-up. Among the 127 children for whom no genotyping data was available, 48 were absent or refused blood sampling and, for the 79 remaining children, technical problems occurred at the time of DNA extraction or DNA quality control. Children for whom DNA was not available were significantly younger than other (5.10 years [SEM = 0.21] and 8.71 years [0.18] respectively; p<10^−3^). However, there was no difference concerning the 4 phenotypes under study between the two groups of children.

Genotyping was done with Affymetrix GeneChip Human Mapping 250K *Nsp* which covers entire genome with ∼262 000 SNPs. Genotyping was performed according to the manufacturer's instructions. Briefly, total genomic DNA was digested with the NspI, ligated to the adaptor, and amplified by polymerase chain reaction (PCR) with a single primer set. After purification of the PCR products, amplicons were quantified, fragmented, labeled, and subsequently hybridized to the 250K SNP mapping array. The genotype of each SNP was determined by the BRLMM algorithm. A call rate (percentage of SNPs genotyped by sample) of 98.6% was obtained across the entire sample. Mapping order, physical and genetic distances of markers were obtained from Affymetrix. Note that physical distances for this GeneChip are based on NCBI Reference Genome Sequence Build 36.3.

Rigorous quality control was performed before statistical analyses to ensure reliable genotyping data. Six samples with a call rate<95% were deleted. Gender of each sample was checked with the number of heterozygosities at SNPs on chromosome X and the relatedness of individuals was analysed using the GRR program [71]. After corrections for pedigree errors, 2 additional samples with no relationship with any of participants were deleted. In the end 372 children of 133 families were included in analysis. The number of children per family ranged from 1 to 7 with a mean number of 2.80 children per family; 374 sib-pairs and 40 half-sib-pairs were available for linkage analysis.

Allele frequencies and tests for Hardy-Weinberg equilibrium (HWE) were calculated from founders. Pedstats [72] was used to detect genotypes with Mendelian inconsistency. SNPs were filtered according to the following parameters: a sample call rate <95%, minor allele frequencies <5% and a deviation from HWE at p-value <10^−4^. Then we examined the relationship between the number of Mendelian errors detected for each SNP and the deviation from HWE. We observed a high inflation of the percentage of SNPs out of HWE for SNPs with more than 8 Mendelian errors, indicating a genotyping of poor quality, and removed 3529 SNPs with more than 8 Mendelian errors. For remaining Mendelian errors, genotypes were deleted in members of the respective families. Non mendelian errors, i.e. unlikely genotype, were also investigated with MERLIN [73] and were automatically removed. In a last step, as we choose to use the method proposed by MERLIN to take into account the LD between SNPs in linkage analysis, we deleted additional 16876 SNPs which were in complete association (r^2^ = 1) with another proximate SNP in our data to avoid large block of SNPs. Exclusion of these SNPs was done using the Tagger tag SNP selection algorithm [74] implemented in Haploview [75]. In the end, analyses were carried out on a set of 174 950 SNPs from autosomal chromosomes and pseudo-autosomal region of X and Y chromosomes.

### Statistical analysis

#### Linkage analysis

We performed two multipoint genome-wide linkage analyses on each phenotype using MERLIN program, a variance components linkage analysis [76] and the regression-based approach [77] implemented in MERLIN-REGRESS. Heritability of phenotypes was estimated from VC analysis.

Dense SNP maps have progressively replaced traditional panels of microsatellite markers for genome-wide linkage analyses because they provide more accurate genotyping and higher information content. However the presence of LD between SNPs is known to increase type I error in non-parametric multipoint linkage analyses, especially when founder genotypes are missing [78], which is the case in our study since 15% of parents are missing. We took this point into account by using the method implemented in MERLIN [79]. MERLIN models the LD between markers by organizing SNPs into clusters which are then treated as multi-allelic markers in analyses. A threshold of pairwise r^2^ = 0.05 was used to join SNPs in clusters. However clusters defined by MERLIN are limited in size (21 SNPs) and the model assumes no LD between clusters. Thus we used a second method in the regions where a linkage peak was identified to check that LD was taken into proper account. This method consists in selecting from the whole SNPs available a subset of SNPs with a minimum of LD before realising linkage analysis. We used MASEL algorithm which selects a subset of SNPs with a minimum of LD (here r^2^<0.05) trying to optimise the number of informative SNPs and the SNP distribution along region [80].

The genome-wide significance of linkage peaks was assessed by 10,000 gene dropping simulations on chromosome 22. This procedure enables to determine how many peaks of similar height might arise by chance conditional on the set of phenotypes being analysed, the marker map and the family structure. Quantitative trait linkage analyses were performed on each of these replicates. Then the average number of linkage peaks per replicate with a LOD score greater than or equal to a given threshold was calculated (peaks were defined as local maxima separated by at least 30 cM). As the genetic length of chromosome 22 is approximately 1/44 of the total length of the autosomal genome, the average number of peaks per replicate on the whole genome was obtained by multiplying the previous average number by 44. Following Lander and Kruglyak [30], a peak was considered as ‘genome-wide significant’ if this number was less than 0.05, and ‘genome-wide suggestive’ if it was less than 1. Additionally for each linkage peak an empirical p-value was computed from 100,000 dropping simulations for the SNP (or cluster of SNPs) with maximum LOD score.

#### Family based association analysis

Finally, we performed an association analysis using FBAT method [81] in the regions of suggestive linkage identified in our study and in 2 others regions, 5q31q33 which has been involved in the control of parasitemia and 10p15 for which a strong evidence for linkage to malaria fever episodes was found [29].

Regions around the maximum LOD score were defined using the 1-LOD support method. For 5q31q33 region, we tested association with SNPs of the whole region from 5q31.1 to 5q33.3 (130,400 Kb–160,000 Kb). For 10p15 region analysis was done on a 11 Mb region (as defined by Timman et al. [29]) from 10pter.

FBAT method was applied to test association in the presence of linkage and we used the approach using the empirical variance-covariance estimator [82]. We tested first for association between each individual SNP and phenotypes. Only additive model was considered. To correct for multiple testing, the effective number of independent tests was assessed for each phenotype using the method of Li and Ji [37] implemented in SNPSpd software [83] and a Bonferroni correction was applied. Then a haplotype analysis was carried out using a sliding window approach with 2 sizes of windows (3 and 5 SNPs).
